# The Homogeneous MADM Methods: Is Trade-Off between Attributes Important?

**DOI:** 10.1155/2022/8629986

**Published:** 2022-08-21

**Authors:** Aref Arman, Hosein Arman, Abdollah Hadi-Vencheh

**Affiliations:** ^1^Department of Management, University of Isfahan, Isfahan, Iran; ^2^Department of Management, Najafabad Branch, Islamic Azad University, Najafabad, Iran; ^3^Department of Mathematics, Isfahan (Khorasgan) Branch, Islamic Azad University, Isfahan, Iran

## Abstract

Compensatory multiattribute decision-making (MADM) methods are founded on the trade-offs between attributes, allowing an alternative to compensate for its weakness in an attribute with its strength in another attribute. We call them heterogeneous MADM methods because they generally consider the unlimited trade-off between attributes. In other words, they even allow that very poor performance of an attribute to be compensated by the strong performance of another attribute. However, this may not be acceptable to decision makers (DMs). They may accept the limited trade-offs between attributes, making them more homogeneous. In these situations, MADM methods should be modified to consider the limited trade-offs between attributes. This modification comes with some conceptual and technical difficulties. This study presents some examples to show the concept of limited trade-offs clearly and presents a modified version of the simple additive weighting (SAW) method, H-SAW, considering the limited trade-offs between attributes. We also integrate H-SAW and fuzzy analytic hierarchy process (FAHP) methods to supplier selection and illustrate the real application of H-SAW method.

## 1. Introduction

Multiattribute decision-making (MADM) methods are generally divided into non-compensatory and compensatory models [1]. Non-compensatory models do not consider the trade-offs between attributes. In these models, each attribute stands independently. Therefore, weakness in an attribute cannot be compensated by the strength of another attribute. Some non-compensatory models are dominance, maximin, maximax, conjunctive, disjunctive, and lexicographic models. For instance, consider the conjunctive (satisficing) method. In this method, the decision maker (DM) determines the minimal values (the cutoff values) of attributes that are acceptable for alternatives. In other words, if an alternative achieves these values, it can be chosen by the DM [1].

In contrast, compensatory models consider the trade-offs between attributes. It means the strength of an attribute can compensate for the weakness of the other attribute. Some conventional compensatory models are simple additive weighting (SAW) method [2], weighted sum model (WSM) [3], weighted product model (WPM) [4], the technique for order preferences by similarity to an ideal solution (TOPSIS) method [1], analytical hierarchy process (AHP) [5, 6], and VlseKriterijumska Optimizacija I Kompromisno Resenje (VIKOR) [7]. We can also mention some newer compensatory models, including the weighted distance-based approximation (WDBA) [8], weighted aggregated sum product assessment (WASPAS) [9], evaluation based on distance from average solution (EDAS) [10], best-worst method (BWM) [11], combinative distance-based assessment (CODAS) method [12], and combined compromise solution (CoCoSo) method [13]. Some studies use different approaches to consider the trade-offs between attributes. For example, Garmabaki et al. [14] formulate a mathematical model based on multiattribute utility theory (MAUT) for this purpose.

Considering unlimited trade-offs between attributes may sometimes be a weakness of compensatory methods. For example, suppose an alternative is exaggeratedly superior to the other alternatives in terms of an attribute but performs very weak in other attributes. A compensatory method may select this alternative as the best one due to the unlimited trade-offs between the attributes. However, the DM does not necessarily agree with this decision. The DM may accept the limited trade-off between attributes, not unlimited. The following example can better illustrate this problem.

Assume that we aim to rank two cell phones that are the same in all features and differ only in price and camera quality. The price and camera quality for the first cell phone are $200 and 20 megapixels (MPs), while these values for the second one are $100 and 10 MPs. These two attributes are equally important to the DM. The most compensatory methods, such as SAW and TOPSIS, assign equal weights to these cell phones. However, the DM does not necessarily accept this result. The DM may accept the limited trade-off between camera quality and price. In other words, the DM may believe that the strength of camera quality should partially compensate for the weakness of price and vice versa. On the one hand, unlimited price increases along with unlimited camera quality increases are not acceptable. On the other hand, unlimited camera quality decreases along with unlimited price decreases are not acceptable. Suppose the DM is unwilling to pay more for camera quality more than 16 MPs. This condition changes the weights of cell phones.

Many real-world problems, such as supplier selection, employ MADM methods to rank the alternatives. For this purpose, researchers have used different MADM methods. TOPSIS is one of the most widely used MADM methods for this purpose. For instance, one can read Kannan et al. [15]; Lee et al. [16]; Fallahpour et al. [17]; Mousakhani et al. [18]; Bai and Sarkis [19]; Jain et al. [20]; Mohammed et al. [21]; Li et al. [22]; Memari et al. [23]; Tirkolaee et al. [24]; Mina et al. [25]; and Kaur and Prakash Singh [26]. The other used common method is VIKOR [27–29]; Abdel-Baset et al. [30]; and Kannan et al. [31]. The other MADM methods have typically been used for supplier selection. We can refer to ANP [32], PROMETHEE [33], ELECTRE-TRI [34], and ARAS [35]. These studies all suffer from a common shortcoming. They apply MADM methods using the unlimited trade-offs between attributes. Therefore, they may select a supplier that performs extraordinarily in some criteria but very poorly in others. Experts do not necessarily agree with this decision. They may prefer to select a supplier coming with acceptable performance for all criteria.

Among different compensatory methods, AHP considers the limited trade-offs between attributes by presenting the homogeneity axiom. According to Saaty [6]; since the mind cannot compare widely disparate elements, they must be homogeneous. AHP considers that the maximum ratio of the importance of two attributes to be 9 and accordingly forms a homogeneous problem. In other words, it compensates for the weakness of an attribute by the strength of another attribute up to a maximum of 9 times. Homogeneity is essential for meaningful comparisons [6]. A comparison matrix in AHP is filled based on two principles: homogeneity and compensability. However, the most compensatory methods are formed based on the decision matrix, which is filled neither based on homogeneity nor limited trade-offs between attributes. Although compensatory methods include steps considering the trade-offs between the decision matrix data, they do not include the steps to consider the homogeneity of alternatives.

This study modifies the SAW method as a compensatory method to consider the homogeneity of alternatives in terms of different criteria. The reason for choosing the SAW method is its simplicity. This worthy to note that the proposed methodology can be extended to other MADM methods, such as TOPSIS and VIKOR, among others. We call the proposed method as homogeneous simple additive weighting (H-SAW) method. The presented method determines the absolute desirable and undesirable thresholds for each attribute. An absolute desirable threshold is an upper (a lower) value for a profit-type (cost-type) attribute so that a part of data that is above (below) this value is not taken into account when trading off between alternatives. On the other hand, an absolute undesirable threshold is a lower (an upper) value for a profit-type (cost-type) attribute so that the data that are smaller (greater) than this value are completely undesirable. The H-SAW method can be considered as a combination of conjunctive and SAW methods. Using SAW or H-SAW to solve a problem depends on the DM. To the best of our knowledge, H-SAW is the only compensatory MADM method using the limited trade-offs between attributes in a decision matrix.

The rest of this paper is organized as follows: Section 2 provides a brief background on SAW and FRSM; Section 3 proposes the H-SAW method; Section 4 gives different examples to illustrate the proposed model; Section 5 concludes and gives suggestions for future research.

## 2. Background

This section is divided into two subsections reviewing the SAW and the fuzzy AHP (FAHP) methods. We review the SAW method because our contribution is based on this method. We also review the FAHP method because we propose a procedure to rank the suppliers by integrating the FAHP and H-SAW methods.

### 2.1. Simple Additive Weighting (SAW) Method

The SAW method is a well-known and widely used MADM methods due to its simplicity. To review this method, consider a decision matrix as

(1) $$\begin{array}{c} D:\begin{array}{ccccc} \; & C_{1} & C_{2} & \; & C_{m}\\ A_{1} & r_{11} & r_{12} & \ldots & r_{1m}\\ \vdots & \vdots & \vdots & \vdots & \vdots \\ A_{n} & r_{n1} & r_{n2} & \ldots & r_{nm} \end{array}, \end{array}$$

where *n* and *m* are the numbers of alternatives and attributes, *A*_*i*_and *C*_*j*_ represent the alternative *i* and the attribute *j*, respectively, and *r*_*ij*_ is the value of alternative *i* for attribute *j*. The SAW method consists of two steps to rank the alternatives described below [1].

**Step 1 .**

Data normalization. This step normalizes the data given in the decision matrix. If *n*_*ij*_ is the normalized value of *r*_*ij*_, it can be obtained as

(2) $$\begin{array}{c} n_{ij}=\left\{\begin{array}{cc} \frac{r_{ij}}{r_{j}^{\max}}, & \text{if }j\in J^{+},\\ \frac{r_{j}^{\min}}{r_{ij}}, & \text{if }j\in J^{-}, \end{array}\right. \end{array}$$

where *J*^+^ and *J*^−^ denote the benefit-type and cost-type sets, respectively, and *r*_*j*_^ max^ and *r*_*j*_^ min^ are the largest and smallest data for attribute *j* in decision matrix (1). Note that some studies obtained the value of *n*_*ij*_ as

(3) $$\begin{array}{c} n_{ij}=\left\{\begin{array}{cc} \frac{r_{ij}-r_{j}^{\min}}{r_{j}^{\max}-r_{j}^{\min}}, & \text{if }j\in J^{+},\\ \frac{r_{j}^{\max}-r_{ij}}{r_{j}^{\max}-r_{j}^{\min}}, & \text{if }j\in J^{-}. \end{array}\right. \end{array}$$

**Step 2 .**

Ranking the alternatives. If *w*_*j*_ (*j* = 1,…, *n*) represents the weight of *j*th attribute, the weight of *i*th alternative (*wA*_*i*_) is obtained as

(4) $$\begin{array}{c} wA_{i}=\sum_{j=1}^{m}w_{j}.n_{ij}. \end{array}$$

The greatest value of *wA*_*i*_ represents the best alternative.

### 2.2. Fuzzy Row Sums Method (FRSM)

FRSM is a FAHP method proposed by Arman et al. [36]. FRSM can be applied to different types of fuzzy numbers. Here, we review this method proposed for triangular fuzzy numbers (TFNs). Consider $\tilde{A}$ as a comparison matrix filled with triangular fuzzy preferences as

(5) $$\begin{array}{c} \tilde{A}={\left({\tilde{a}}_{ij}\right)}_{n\times n}=\left[\begin{array}{cccc} \left(1,1,1\right) & \left(l_{12},m_{12},u_{12}\right) & \ldots & \left(l_{1n},m_{1n},u_{1n}\right)\\ \left(l_{21},m_{21},u_{21}\right) & \left(1,1,1\right) & \ldots & \left(l_{2n},m_{2n},u_{2n}\right)\\ \vdots & \vdots & \vdots & \vdots \\ \left(l_{n1},m_{n1},u_{n1}\right) & \left(l_{n2},m_{n2},u_{n2}\right) & \ldots & \left(1,1,1\right) \end{array}\right], \end{array}$$

where *n* is the number of elements, and ${\tilde{a}}_{ij}=\left(l_{ij},m_{ij},u_{ij}\right)={\tilde{a}}_{ji}^{-1}=\left(1/u_{ji},1/m_{ji},1/l_{ji}\right).$ FRSM extracts the local weights from this matrix using the following steps.

Step 1. Sum up each row of the matrix *l*_*i*_ as
  (6) $$\begin{array}{c} RS_{i}=\sum_{j-1}^{n}\tilde{a_{ij}}=\left(\sum_{j=1}^{n}l_{ij},\sum_{j=1}^{n}m_{ij},\sum_{j=1}^{n}u_{ij}\right),i=1,\ldots ,n, \end{array}$$
where *RS*_*i*_ is the sum of TFNs in row *i*.
Step 2. Normalize *RS*_*i*_ through
  (7) $$\begin{array}{c} {\tilde{S}}_{i}=\frac{RS_{i}}{\sum_{j-1}^{n}RS_{j}}=\left(\frac{\sum_{j-1}^{n}l_{ij}}{\sum_{j-1}^{n}l_{ij}+\sum_{\begin{array}{c} k-1\\ k\neq i \end{array}}^{n}\sum_{j-1}^{n}u_{kj}},\frac{\sum_{j-1}^{n}m_{ij}}{\sum_{k-1}^{n}m_{kj}},\frac{\sum_{j-1}^{n}u_{ij}}{\sum_{j-1}^{n}u_{ij}+\sum_{\begin{array}{c} k-1\\ k\neq i \end{array}}^{n}\sum_{j-1}^{n}l_{kj}}\right),i=1,\ldots ,n, \end{array}$$
where ${\tilde{S}}_{i}$ is the fuzzy local weight of the element corresponding to row *i*; this weight is shown as ${\tilde{S}}_{i}=\left(l_{{\tilde{S}}_{i}},m_{{\tilde{S}}_{i}},u_{{\tilde{S}}_{i}}\right)$ and can be approximately considered a TFN.
Step 3. Defuzzify ${\tilde{S}}_{i}$ to obtain the crisp local weights. Arman et al. [36] showed that ${\tilde{S}}_{i}$ can be defuzzified as
  (8) $$\begin{array}{c} S_{i}=\frac{l_{{\tilde{S}}_{i}}+m_{{\tilde{S}}_{i}}+u_{{\tilde{S}}_{i}}}{3},\;i=1,...,n. \end{array}$$
Using the center of gravity method.
Step 4. The sum of the defuzzified local weights obtained in Step 3 is not necessarily equal to 1. Therefore, normalize these weights as
  (9) $$\begin{array}{c} w_{i}=\frac{\sum_{i=1}^{n}S_{i}}{n}, \end{array}$$
where *w*_*i*_ is the crisp local weight of element *i*.

## 3. Homogeneous Simple Additive Weighting (H-SAW) Method

In this section, we modify the SAW method to consider the limited trade-offs between the attributes. Consider the decision matrix (1) in which the data of *n* alternatives are given for *m* attributes. Here, we present the H-SAW method to rank the alternatives. The presented method consists of three steps as follows.

Step 1. Determining the thresholds. This step extracts the desirable and undesirable thresholds for each attribute using the experts' opinions. Let *J*^+^ and *J*^−^ be the profit- and the cost-type attribute sets, respectively. If the attribute *j* belongs to *J*^+^, its desirable and undesirable thresholds are shown as *U*_*j*_^+^ and *L*_*j*_^+^, respectively. If the experts do not determine the thresholds for the benefit-type attribute *j*, these values can be obtained as
  (10) $$\begin{array}{c} \text{Desirable threshold}:U_{j}^{+}=r_{j}^{\max},j\in J^{+}\\ \text{Undesirable threshold}:L_{j}^{+}=r_{j}^{\min},j\in J^{+}. \end{array}$$
On the other hand, if the attribute *j* belongs to *J*^−^, its desirable and undesirable thresholds are shown as *L*_*j*_^−^ and *U*_*j*_^−^, respectively. If the experts do not determine the thresholds for the cost-type attribute *j*, these values can be obtained as
  (11) $$\begin{array}{c} \text{Desirable threshold}:L_{j}^{-}=r_{j}^{\min},j\in J^{-}\\ \text{Undesirable threshold}:U_{j}^{-}=r_{j}^{\max},j\in J^{-}. \end{array}$$
Step 2. Homogeneous normalization. This step obtains *n*_*ij*_ as the homogeneous normalized value of *r*_*ij*_. If the attribute *j* belongs to *J*^+^, the normalized value of *r*_*ij*_ is obtained as
  (12) $$\begin{array}{c} n_{ij}=\left\{\begin{array}{cc} 0, & \text{if }r_{ij}\leq L_{j}^{+},\\ \frac{r_{ij}-L_{j}^{+}}{U_{j}^{+}-L_{j}^{+}} & \text{if }L_{j}^{+}<r_{ij}<U_{j}^{+}\;\forall_{j\in J^{+}},\\ 1, & \text{if }r_{ij}\geq U_{j}^{+}. \end{array}\right.. \end{array}$$
According to (12), the homogeneous normalized value for all data greater than or equal to *U*_*j*_^+^ equals 1. In other words, (12) does not allow a part of data over *U*_*j*_^+^ to be considered when trading off between attributes. Also, the homogeneous normalized value for all data less than or equal to *L*_*j*_^+^ is 0 using this equation. It means that all data less than *L*_*j*_^+^ for attribute *j* are ignored by experts when evaluating the alternatives.  Figure 1(a) shows the normalized value for a profit-type attribute schematically.
On the other hand, if the attribute *j* belongs to *J*^−^, the homogeneous normalized value of *r*_*ij*_ is obtained as
  (13) $$\begin{array}{c} n_{ij}=\left\{\begin{array}{cc} 0, & \text{if }r_{ij}\geq U_{j}^{-},\\ \frac{U_{j}^{-}-r_{ij}}{U_{j}^{-}-L_{j}^{-}} & \text{if }L_{j}^{-}<r_{ij}<U_{j}^{-}\;\forall_{j\in J^{-}},\\ 1, & \text{if }r_{ij}\leq L_{j}^{-} \end{array}\right.. \end{array}$$
(13) assigns the homogeneous normalized value of 1 to all data smaller than or equal to *L*_*j*_^−^. This causes that all data less than *L*_*j*_^−^ to have the same importance when trading off between attributes. Also, the homogeneous normalized value for all data greater than or equal to *U*_*j*_^−^ is 0 using this equation. It means that all data greater than *U*_*j*_^−^ for attribute *j* is completely undesirable, according to experts. Note that (13) converts an original disutility data into a utility value. In other words, *r*_*ij*_ is a disutility data, i.e., the less, the better; however, *n*_*ij*_ is a utility value, i.e., the more, the better.  Figure 1(b) shows the schematic of a normalized value for a cost-type attribute.
Step 3. Ranking the alternatives
If *w*_*j*_ (*j* = 1,…, *n*) is the weight of *j*^*th*^ attribute, the final weight of *i*^*th*^ alternative (*wA*_*i*_) is obtained as
  (14) $$\begin{array}{c} wA_{i}=\sum_{j=1}^{m}w_{j}.n_{ij}. \end{array}$$
The alternatives are ranked based on *wA*_*i*_ ascendingly. Therefore, the best alternative is obtained as
  (15) $$\begin{array}{c} A^{*}=\left\{\frac{A_{i}|\max\;\sum_{j=1}^{n}w_{j}n_{ij}}{\sum_{j=1}^{n}w_{j}}\right\}. \end{array}$$

Note. MADM methods improve the decision-making process by decomposing the overall assessment of alternatives to the assessment of a number of often conflicting criteria [37]. In other words, a user can go through iterations to rank the alternatives in an MADM method [38]. These iterations, which can be shown as a flowchart, increase the clarity of an MADM algorithm. For this reason, here, we present the flowchart of H-SAW method (Figure 2).

## 4. Application

In this section, we use two different examples to show the applications of the H-SAW method.

**Example 1 .**

This example uses the hypothetical data and aims to rank three cell phones (*A*_*1*_, *A*_*2*_, and *A*_*3*_) considering two attributes: the price (*C*_*1*_) and the camera quality (*C*_*2*_). The data relating to these attributes for three cell phones are given in Table 1. If the weights of price and camera quality are 0.4 and 0.6, respectively, SAW selects *A*_*1*_ as the best alternative. The related calculations are given in Table 1.

Now assume that the DM would not pay more for the camera quality of more than 16 MPs. In other words, the high camera quality of more than 16 MPs for a cell phone to compensate for the high price of that cell phone is not acceptable to experts. On the other hand, the camera quality less than or equal to 12 MPs comes with the satisfaction of 0. Also, the DM want not to pay the price of less than $120 to compensate for the low camera quality. On the other hand, a price greater than or equal to $170 is completely undesirable for the DM. According to these explanations, the normalization functions for camera quality and price can be shown in Figures 3(a) and 3(b), respectively.

The H-SAW selects *A*_*2*_ as the best alternative. The related calculations are given in Table 2.

Comparing Tables 1 and 2 shows that SAW selects *A*_*1*_ as the best alternative, while H-SAW selects *A*_*2*_ as the best one. This example shows that the limited trade-offs between attributes can significantly change the ranking of alternatives.

**Example 2 .**

This example presents a real case in which the suppliers are ranked with respect to the supply chain risks of a steel company. According to experts, the risks related to supplying the graphite electrode are the most critical. Graphite electrode is the conducting element for electric arc furnaces steelmaking. The most critical risks that may occur in the future when supplying the graphite electrode includes:

1. Graphite electrode price rise (*R*_1_)
2. Non-flexibility in supply capacity (*R*_2_)
3. The order deliverance delay (*R*_3_)
4. Low-quality of the graphite electrode (*R*_4_)

There are four main suppliers of graphite electrodes. We rank them considering the different risks of graphite electrodes. For this purpose, we follow three phases. Phase 1 obtains the weights of these risks based on the experts' opinions. Phase 2 extracts the homogeneous normalization functions for different risks. Phase 3 uses the H-SAW to rank the suppliers. These phases are described in detail as follows.

**Phase 1 .**

Obtaining the weights of risks

In this phase, we obtain the weights of four risks related to supplying the graphite electrode. For this purpose, we provide a pairwise comparison matrix and arrange a panel of experts to fill this matrix. This matrix is filled by the relative linguistic preferences based on the experts' consensus and then replaced by their equivalent TFNs according to Table 3.

Therefore, we form a fuzzy comparison matrix based on the experts' opinions (Table 4).

We use the FRSM to extract the crisp local weights from this matrix. The related computations are given in Table 5.

Table 5 depicts that the non-flexibility in supply capacity (*R*_2_) is the most critical risk that the company may face in the future when supplying the graphite electrode.

**Phase 2 .**

Extracting the homogeneous normalization functions

This section first forms a decision matrix and then extracts the homogeneous normalization functions for different risks.  Table 6 represents the suppliers' data for each risk. This table also gives the desirable and undesirable values for each attribute. These values are obtained from the experts' opinions. Due to company considerations, the data related to each attribute are multiplied by a positive number. Therefore, the values in Table 6 do not represent the real data. However, these changes do not affect the supplier ratings because of the normalization step.

In the following, we extract a homogeneous normalization function for each risk.

The homogeneous normalization function of price. Prices are estimated for the future period, according to experts. The experts do not determine the thresholds for price because the lower (higher) the price is, the more favorable (unfavorable) it is. Therefore, we define the desirable and undesirable thresholds for price using (11), i.e., 685 and 889, respectively. Price is a cost-type attribute. Therefore, different suppliers' prices should be normalized using the following equation:

(16) $$\begin{array}{c} n_{i1}^{\text{Price}}=\left\{\begin{array}{cc} 0, & \text{if }r_{i1}\geq 889,\\ \frac{889-r_{i1}}{889-685}, & \text{if }685<r_{i1}<889,\\ 1, & \text{if }r_{i1}\leq 685. \end{array}\right. \end{array}$$

The homogeneous normalization function of coverage. Excess demand coverage (in percent) is an attribute related to the risk of non-flexibility in supplier capacity. Experts estimate the company will need more graphite electrodes in the next period. This surplus of demand is about 32% more than the current consumption. They also estimate the percent of this excess demand that each supplier can cover. It is clear that a supplier's potential to provide graphite electrodes above 32% is not advantageous for that supplier from the company's perspective. On the other hand, a supplier's potential to cover the excess demand of less than 15% is not favorable to experts because it will probably force the company to buy from different suppliers, leading to a high supplying cost. Therefore, the desirable and undesirable thresholds for excess demand coverage are 32% and 15%, respectively. Excess demand coverage is a benefit-type attribute. Therefore, its different values should be normalized using the following equation:

(17) $$\begin{array}{c} n_{i2}^{\text{Coverage}}=\left\{\begin{array}{cc} 0, & \text{if }r_{i2}\leq 15,\\ \frac{r_{i2}-15}{32-15}, & \text{if }15<r_{i2}<32,\\ 1, & \text{if }r_{i2}\geq 32. \end{array}\right. \end{array}$$

The homogeneous normalization function of delay. Experts estimate order deliverance delay (in days) for each supplier based on their experience. If the delay is more than 30 days, it is not acceptable for the company because it causes uncertainty that forces the company to buy and store more graphite electrodes. On the other hand, a delay of fewer than 14 days does not make an advantage for suppliers to compensate for their unfavorable attributes because the company stores enough graphite electrodes as a safety stock that meets the need for at least 14 days. It means the desirable and undesirable thresholds for delay are 14 and 30 days, respectively. Delay is a cost-type attribute. It means the equation that normalizes different suppliers' delays is formed as

(18) $$\begin{array}{c} n_{i3}^{\text{Delay}}=\left\{\begin{array}{cc} 0, & \text{if }r_{i1}\geq 30,\\ \frac{30-r_{i1}}{30-14} & \text{if }14<r_{i1}<30,\\ 1, & \text{if }r_{i1}\leq 14. \end{array}\right. \end{array}$$

The homogeneous normalization function of quality. Experts assess the quality of graphite electrodes produced by each supplier. There are different measures to determine the quality of graphite electrodes, including their diameters, resistivity, bulk density, bending strength, and petroleum coke grades. We ask the experts to estimate the quality of the graphite electrode produced by each supplier. For this purpose, the experts' opinions are extracted using a multiple-choice questionnaire as linguistic terms, which are then converted to the crisp scores according to Table 7.

Different experts have different opinions. Therefore, we calculate the average of the experts' scores for each supplier as its final score for quality attribute, given in Table 6. Experts believe that all quality scores less than 1.5 are not desirable because they impose almost an equal extra cost to the company. On the other hand, the experts believe that the quality score in excess of 3.5 is not the advantage of the suppliers and should not be considered to compensate for the suppliers' weakness in other attributes. As a result, the desirable and undesirable thresholds for quality scores are 3.5 and 1.5, respectively. Quality is a benefit-type attribute. Therefore, its different values are normalized using the following equation:

(19) $$\begin{array}{c} n_{i4}^{\text{Quality}}=\left\{\begin{array}{cc} 0, & \text{if }r_{i4}\leq 1.5,\\ \frac{r_{i4}-1.5}{3.5-1.5}, & \text{if }1.5<r_{i4}<3.5,\\ \; & \text{if }r_{i4}\geq 3.5. \end{array}\right.. \end{array}$$

**Phase 3 .**

Ranking the suppliers

Here, we use the H-SAW method to rank the suppliers considering the graphite electrode risks. For this purpose, first, we normalize the data given in Table 6 using the normalizing functions presented in Phase 2. The results are given in Table 8. This table also gives the weights of attributes obtained in Phase 1. Therefore, the weights of suppliers are calculated using (14), and accordingly, the suppliers are ranked. These results are shown in Table 8.

## 5. Discussion and Conclusion

The hybrid approach of MADM techniques is one of the approaches used by researchers to rank the suppliers. One of the most commonly used hybrid strategies for this purpose is to combine the AHP and TOPSIS methods. AHP is typically used to weigh the criteria, and TOPSIS ranks the suppliers. Lee et al. [16]; Jain et al. [20]; Mohammed et al. [21]; and Mina et al. [25] used this strategy to rank the suppliers. Researchers also used the other combinations for this purpose. For example, Kuo et al. [27] used a hybrid approach consisting of an analytic network process (ANP) and VIKOR to rank the green suppliers. Abdel-Baset et al. [30] used a hybrid approach based on ANP and VIKOR to rank the sustainable suppliers. Fu [35] integrated AHP with ARAS to rank the suppliers. Guarnieri and Trojan [34] evaluated the performance of suppliers using AHP and ELECTRE-TRI methods.

Some of the mentioned studies applied a combination of fuzzy MADM methods to rank the suppliers. We can also refer to other fuzzy combination approaches proposed for this purpose. For example, Prasanna Venkatesan and Goh [33] ranked the suppliers using a hybrid fuzzy AHP and PROMETHEE methods. Valipour Parkouhi and Safaei Ghadikolaei [28] combined fuzzy ANP (FANP) and gray VIKOR to rank the suppliers in a resilient framework. Awasthi et al. [29] obtained the weights of criteria using FAHP and then selected the suppliers using the fuzzy VIKOR. Kannan et al. [31] selected the sustainable suppliers by the combination of fuzzy BWM and interval VIKOR. Tirkolaee et al. [24] applied the FANP to weight the criteria and then used fuzzy TOPSIS to prioritize the suppliers.

Among the various MADM methods, AHP and ELECTRE III consider limited trade-offs between attributes. However, these methods come with some disadvantages that H-SAW avoid. ELECTRE III is the most superior outranking methodology as it uses thresholds for modeling imprecise data [39]. It considers three threshold values for each criterion: indifference, preference, and veto. Using this method may cause that very poor performance on a single criterion eliminates an alternative from consideration. Also, its algorithm is relatively complex and may not be understood by the decision maker. Using ELECTRE III also may not necessarily lead to a complete ranking of alternatives [40].

The advantageous of AHP is the availability of user-friendly and commercially supported software packages [41]. Also, pairwise comparisons provide an uncomplicated way to enter qualitative preferences. However, AHP suffer from some disadvantages, including the possibility for intransitive preferences, high number of pairwise comparisons required for large-scale problems, and an inherent flaw termed rank reversals that occur when an alternative is added or removed from a decision model after preferences [40]. It also suffers from uneven dispersion of values in Saaty's AHP selection scale. In other words, the difference in selecting between the scale of 1 and 2 is about 15 times greater than the difference in selecting between the scale of 8 and 9 [42]. Moreover, AHP analysis is comparatively time-consuming and cumbersome because it requires many pairwise comparisons [40]. This disadvantageous is more highlighted when the number of elements in a pairwise comparison matrix (*n*) increases because the number of required pairwise comparisons is 1/2*n*(*n* − 1).

Some other studies compared different MADM methods under fuzzy environment. In this field, Zamani-Sabzi et al. [43] applied different triangular fuzzy MADM methods on the same decision matrices and then computed the Kendall's tau-b correlation coefficients between them. The results showed that fuzzy SAW, TOPSIS, WPM, and AHP have statistically similar performances; fuzzy ELECTRE is not preferable in providing full and sorted ranks among the alternatives; fuzzy VIKOR may categorizes several alternatives with the same ranks and therefore it is unfavorable technique when full and sorted ranks are required. The results also showed that some methods like fuzzy SAW and TOPSIS are computationally simple to apply, while some others like fuzzy ELECTRE, VIKOR, and AHP are computationally large and elaborate. Zamani-Sabzi et al. [43] showed that simple fuzzy MADM methods under fuzzy environment match the performance of complicated MADM methods; thus, in comparison with the other evaluated methods, they concluded that fuzzy SAW can be an especially simple method to understand and apply in ranking the alternatives of a decision matrix. Based on these expressions, we decided to present homogeneous version of SAW method in this study.

In this study, we applied a new hybrid approach of MADM methods to rank the suppliers. Our approach differs from similar approaches in different aspects. Firstly, we ranked the suppliers based on the possible risks that they may occur in the future. For this purpose, we used the experts' knowledge about the suppliers and their possible performance in the future. This approach contrasts with those ranking the suppliers based on their past performance. Secondly, we obtained the weights of these risks using a new FAHP method proposed by Arman et al. [36]. They first discussed in their study that the existing FAHP methods suffer from different shortcomings and then presented four approximated FAHP methods to avoid them.

Thirdly, we ranked the suppliers using the H-SAW method. This is the most important difference between our approach and similar approaches in supplier selecting. The other studies suffer from a common shortcoming. They apply MADM methods using the unlimited trade-offs between attributes. Therefore, a supplier may be selected as the best one with extraordinary performance in some criteria but poor performance in others. For example, MADM methods may select a supplier as the best one, with outstanding performance in deliverance but very low-quality material. The reason for this selection is that the outstanding performance in deliverance unlimitedly can compensate for the very poor quality of materials. However, experts may prefer to select a supplier with acceptable performance for all criteria. H-SAW method, presented in this study, avoids unlimited trade-offs between attributes when evaluating the suppliers.

As a modification of the SAW method, the H-SAW method restricts the trade-offs between attributes. Unlike the SAW method, H-SAW does not allow the very poor performance of an attribute to be fully compensated by the strong performance of other attributes. For this purpose, it determines an upper (a lower) value for a benefit (cost) type attribute as its desirable threshold. This value can be obtained from the experts' opinions. H-SAW does not consider a part of the data that is greater (smaller) than the desirable threshold when trading off between attributes. This is conceptually similar to the homogeneity axiom of AHP. According to this axiom, each attribute is allowed to be up to 9 times preferable to other attributes. In other words, no matter how much the preference of two attributes is greater than 9, AHP does not consider a part of this preference that exceeds 9. Using the SAW or H-SAW methods in a real situation depends on the experts.

In this study, we presented the H-SAW method based on the homogeneous normalization functions. We defined these functions similarly to the membership functions in fuzzy sets. Future research could use other approaches to derive homogeneous normalization functions. It is also suggested that the homogeneous versions of other compensatory MADM methods are presented. Therefore, we expect future research to present other homogeneous MADM methods, including the homogeneous TOPSIS and homogeneous VIKOR.

## Figures and Tables

**Figure 1:** The schematics of homogeneous normalization functions. (a) Benefit-type attribute (b) cost-type attribute.

**Figure 2:** The H-SAW algorithm.

**Figure 3:** The schematics of homogeneous normalizing. (a) The camera quality attribute (b) the price attribute.

**Table 1:** The related calculations for the SAW method.

Alternatives	The original data		The normalized values		Weights of alternatives	Rankings
	*C*_1_	*C*_2_	*C*_1_	*C*_2_		
A_1_	200	20	0.5	1	0.80	1
A_2_	160	16	0.625	0.8	0.73	2
A_3_	100	10	1	0.5	0.70	3
Weights of attributes			0.4	0.6		

**Table 2:** The related calculations for the H-SAW method.

Alternatives	The original data		The normalized values		Weights of alternatives	Rankings
	*C*_1_	*C*_2_	*C*_1_	*C*_2_		
A_1_	200	20	0	1	0.60	2
A_2_	160	16	0.2	1	0.68	1
A_3_	100	10	1	0	0.4	3
Weights of attributes			0.4	0.6		

**Table 3:** Linguistic preferences and their equivalent TFNs.

Definitions	Row to column preference	Column to row preference
Equal importance	(1, 1, 1)	(1, 1, 1)
Equal to relatively more important	(1, 2, 3)	(0.333, 0.5, 1)
Relatively more important	(1, 3, 5)	(0.2, 0.333, 1)
Relatively important to high importance	(3, 4, 5)	(0.2, 0.25, 0.333)
High importance	(3, 5, 7)	(0.143, 0.2, 0.333)
High importance to very high importance	(5, 6, 7)	(0.143, 0.167, 0.2)
Very high importance	(5, 7, 9)	(0.111, 0.143, 0.2)
Very high importance to completely important	(7, 8, 9)	(0.111, 0.125, 0.143)
Completely important	(7, 9, 9)	(0.111, 0.111, 0.143)

**Table 4:** The fuzzy comparison pairwise of graphite electrode risks.

Risks	*R*_1_	*R*_2_	*R*_3_	*R*_4_
*R*_1_	(1, 1, 1)	(0.143, 0.2, 0.333)	(0.333, 0.5, 1)	(0.333, 0.5, 1)
*R*_2_		(1, 1, 1)	(1, 2, 3)	(3, 4, 5)
*R*_3_			(1, 1, 1)	(1, 2, 3)
*R*_4_				(1, 1, 1)

**Table 5:** Extracting the weights of graphite electrode risks using FRSM.

Risks	Row sum using equation (6)	Normalizing using equation (7)	Defuzzifying using equation (8)	Crisp weights using equation (9)
*R*_1_	(1.809, 2.2, 3.333)	(0.058, 0.094, 0.194)	0.115	0.110
*R*_2_	(8, 12, 16)	(0.324, 0.512, 0.676)	0.504	0.482
*R*_3_	(3.333, 5.5, 8)	(0.119, 0.235, 0.393)	0.249	0.238
*R*_4_	(2.533, 3.75, 5.333)	(0.085, 0.160, 0.289)	0.178	0.170
Summation			1.046	1

**Table 6:** Decision matrix.

Suppliers	Price	Coverage (the excess demand)	Delay (in order deliverance)	Quality
Supplier 1	712	12	20	1.25
Supplier 2	784	26	28	1.73
Supplier 3	685	9	11	2.92
Supplier 4	889	51	41	3.87
Desirable thresholds	685	32	14	3.5
Undesirable thresholds	889	15	30	1.5

**Table 7:** The linguistic terms and their corresponding crisp values.

Linguistic term	Very low	Low	Medium	High	Very high
Crisp score	1	2	3	4	5

**Table 8:** Supplier selection using the H-SAW method.

Suppliers	Price	Excess demand coverage	Order deliverance delay	Quality	Supplier weights	Supplier rankings
Supplier 1	0.868	0	0.625	0	0.244	4
Supplier 2	0.515	0.647	0.125	0.115	0.418	3
Supplier 3	1	0	1	0.710	0.469	2
Supplier 4	0	1	0	1	0.652	1
Attribute weights	0.110	0.482	0.238	0.170		

## Data Availability

All data used to support the findings of the study are included within the article.
